# Combined application of zinc-lysine chelate and zinc-solubilizing bacteria improves yield and grain biofortification of maize (*Zea mays* L.)

This article has been retracted.

**DOI:** 10.1371/journal.pone.0254647

**Published:** 2021-07-13

**Authors:** Safdar Bashir, Abdul Basit, Rana Nadeem Abbas, Shahbaz Naeem, Saqib Bashir, Niaz Ahmed, Muhammad Saeed Ahmed, Muhammad Zahaib Ilyas, Zubair Aslam, Saqer S. Alotaibi, Ahmed M. El-Shehawi, Yunzhou Li

**Affiliations:** 1 Department of Soil and Environmental Sciences, Ghazi University, Dera Ghazi Khan, Pakistan; 2 Department of Plant Pathology, College of Agriculture, Guizhou University, Guiyang, Guizhou of China; 3 Department of Agronomy, University of Agriculture Faisalabad, Faisalabad, Pakistan; 4 Department of Soil Science, Faculty of Agricultural Sciences and Technology, Bahauddin Zakariya University, Multan, Punjab-Pakistan; 5 Department of Biotechnology, College of Science, Taif University, Taif, Saudi Arabia; Mendel University of Agriculture and Forestry: Mendelova univerzita v Brne, CZECH REPUBLIC

## Abstract

Malnutrition a health disorders arising due to over or low use of minerals, vitamins and nutritional substances required for proper functioning of body tissues and organs. Zinc (Zn) is the most important mineral required for the normal metabolism of plants and humans. Zinc-deficiency is one of the major cause of malnutrition globally. Maize is highly susceptible to Zn-deficiency and inflicts Zn-deficiency to humans and other animals being nourished on it. This study evaluated the effect of zinc-lysine chelate alone (0.1, 0.5, 1.0 and 1.5%) as seed priming and in combination with Zn-solubilizing bacteria (PMEL-1, PMEL-48, PMEL-57and PMEL-71)) on grain biofortification of autumn maize. The Zn accumulation in different parts (roots, stem, leaves, grains and cob pith) was quantified. Results indicated that Zn contents were 18.5% higher in the seeds primed with 1.5% solution of Zn-lysine chelate and inoculation of ZSB strains compared to control treatments. Seed priming with 1.5% Zn-lysine chelate in combination with ZSB inoculation significantly improved cob diameter and cob length by 16.75% and 42% during 2016 and by 11.36% and 34.35% during 2017. The increase in 100 grains weight over control was 18.4% and 15.27% for 2016 and 2017, respectively. The Zn contents were increased by 15.3%, 15.6%, 49.1%, and 33.0% in grain, cob-pith, stemand roots, respectively compared from control. Thus, the combined application of 1.5% Zn-lysine chelates along with ZSB inoculation could be used for combating malnutrition.

## Introduction

Global population is increasing with annual growth rate of 1.03% and 1.95% in Pakistan. According to the estimation of “World Nations”, global population will grow to 8.5 billion in 2030, 9.7 billion in 2050 and 10.9 billion during 2100 [1]. Thus, food demand will also increase and it would be challenging to fulfill global food demands. Yang et al. [2] presented a national survey report showing that 50% people of China suffer from Zn-deficiency. Latest publication of “The State of Food Security and Nutrition in the World” has established a regular checkup for the desired targets set by 2030 agenda regarding food security and nutrition targets [3]. The Zn-deficiency is awide spread problem in Pakistani soils. The 21–77% of the soils in Khyber Pakhtunkhwa (KPK) province are Zn-deficit. Likewise, 42% of agricultural soils in Mansehra and Swat districts of KPK have been declared Zn-deficient [4].

Zinc is an essential micronutrient and required by all organisms [5, 6]. It is required as cofactor for >300 enzymes Coleman [7], and takes part in the structural component of many proteins containing several transcription factors [8, 9]. More than 25% of global human population suffers from Zn-deficiency [10]. In World Health Organization report of 2012, Zn-deficiency was declared 5^th^ among crucial factor of health risks in the developing countries. The Zn-deficiency is important Fe and vitamin-A deficiencies. Grains enriched with Zn can significantly improve health. Moreover, proper Zn nutrition improves crop productivity [11].

Rice-wheat cropping system is practiced on 85% area of south Asia, which is Zn-deficient [12]. Zinc is involved in different mechanisms, including respiration, chlorophyll biosynthesis and photosynthesis; thus, considered more important than other nutrients [13, 14]. About 30% of soils are Zn deficient worldwide [15, 16]. Nonetheless, ~70% of arable lands in Pakistan are deficient [17].

Micronutrient deficiency is an emerging issue in developing and regarded as hidden hunger. Poor health, mental dysfunction and impaired immune system are some of the issues caused by Zn-deficiency. Zinc deficiency is a widespread cause of children’s death throughout the world [18]. Zinc deficiency is common in the countries where cereals are consumed for daily calories and protein [18] and Zn-deficiency was realized as plant nutritional problem throughout rice growing countries such as Japan, USA, Brazil, and Phillipines. Human nutrition and crop productivity can be improved by adding as zinc lysine chelate and zinc solubilizing bacteria to plants. Seed germination under sub-optimal conditions, seed vigor, viability and stand establishment are improved with higher Zn contents in the seeds. Different soil factors are linked with Zn-deficiency, which include high pH, high salinity, high calcium and bicarbonates, waterlogging, intensive cultivation and higher nutrient uptake [19, 20]. Morgan and Drew used the term “chelate” for the compounds capable for the compounds producing complexes with metals that can be used as additives in human and animal nutrition [21]. In 1950s, iron (Fe) chelates were used for the first time to ameliorate Fe-deficiency in plants [22]. Iron amino acid was the first evolved chelate, which was used to improve Fe concentrations in biological systems of human and animals [21]. Foliar application of amino acid chelate with certain Zn-amino chelate increased Zn contents, yield and grain quality of wheat [23]. Several amino chelates are available now, which supply a wide range of nutrients through seeds or foliar application [21].

Although several studies reported that foliar application of Zn improves growth and productivity of maize, very little is known about the impact of Zn seed priming on growth and productivity of maize crop. The available Zn in soil is important for growth of plants; however, Zn uptake is hindered due to its fixation in the soil. The Zn-solubilizing bacteria (ZSB) are capable of enhancing Zn uptake; however, limited studies have been conducted to evaluate the impact of ZSB on Zn uptake in cereals. Therefore, current study was conducted to evaluate the impact of zinc-lysine chelate seed priming in combination with ZSB on Zn availability, uptake and grain biofortification of maize.

## Materials and methods

### Experimental site and soil analysis

The experiments were conducted at Research Farm, Department of Agronomy, University of Agriculture, Faisalabad during autumn, 2016 and 2017. Collected soil samples were analyzed for different physicochemical properties and Zn contents. Faisalabad is situated between 30.35–31.47^o^N latitude, 72.08-73^o^E longitude and 150 m above sea level.

### Physicochemical properties of soil

Soil samples were collected before sowing and after harvesting through standard methods. Soil samples were collected from 0–20 cm depth with soil auger. The total five soil samples were taken from 0–20 cm depth, and they were made composite sample. The samples were packed in polythene bags and transferred to the laboratory. Experimental soil was loamy in nature. Soil properties are summarized in Table 1. Zinc was determined by using Atomic Absorption Spectrophotometer (Hitachi Polarized Zeeman AAS, Z-8200, Japan).

**Table 1:** Physicochemical properties of soil.

Soil property	Before sowing	After harvesting	Before sowing	After harvesting
	2016		2017	
pH	7.4	7.3	7.4	7.4
Electrical Conductivity (EC) (dSm^-1^)	1.54	1.46	1.62	1.45
Organic Matter (%)	1.22	1.28	1.19	1.26
Saturation (%)	32	31	34	32
Phosphorus (ppm)	12.2	9.8	11.5	9.3
Potassium (ppm)	240	224	260	220
Textural analysis	Sand = 40.3, Silt = 32.4, Clay = 27.3			
Zn (ppm)	0.26	0.38	0.28	0.34

### Experimental material

The seeds of maize hybrid 30Y87 (Pioneer) were collected from local grain market, Dijkot Road, Faisalabad. Zinc-lysine chelate was collected from Dr. Muhammad Qasim Associate Professor, Department of Botany, Govt. College University Faisalabad, while zinc solubilizing bacterial strains were isolated in Plant and Microbial Ecology Laboratory, Department of Agronomy, University of Agriculture, Faisalabad, Pakistan.

### Screening of Zn-solubilizing bacteria

For isolation of Zn-solubilizing bacteria, soil samples were taken from the experimental site. The total five soil samples were taken from 0–20 cm depth and they were made composite sample. One gram of soil was added to 10 ml of 50 mM phosphate buffer (pH 7.0) and 50% of the soil mixture was treated by sonication with an electronic homogenizer (Bandelin Sonoplus, Berlin, Germany) at 260 W/cm^2^ for 15 secs to isolate bacteria. Serial dilutions were performed after mixing both sonicated and non-sonicated portions. The diluted aliquots were spread on modified half-strength R2A agar plates [24]. A 100 μl aliquot was applied to half-strength R2A agar medium in large polystyrene Petri dishes (15 cm diameter) for 10^−3^ and10^-5^dilutions, and the plates were incubated at 28°C for 72 hours. The isolation medium was supplemented with 40% (v/v) soil extract and 50 μg/ml amphotericin B to inhibit fungal growth. The colonies were selected based on morphology, and the isolates were sub-cultured on modified half-strength R2A agar plates.

Out of 26 strains, only 4 (PMEL-1, PMEL-48, PMEL-57, and PMEL-71) were selected on the basis of their Zn solubilizing ability and success for 16S rRNA sequencing.

### Seed priming and bacterial inoculation

The maize seeds were primed with different concentrations of Zn-lysine chelate solutions (0.1%, 0.5%, 1.0% and 1.5%) for 10 hr and surface dried for one hour in the laminar flow cabinet (to avoid bacterial contamination) to their original weight. In other treatments 4ZSB strains (PMEL-1, PMEL-48, PMEL-57and PMEL-71) were used. These strains were identified based on 16S rRNA gene sequencing. Seed inoculation was done with standard method [24]. Briefly, seeds were washed twice with ethanol and subsequently with pure distilled water and dried to original weight. Sugar solution (10%) was applied to seed surface as sticky material and carbon source for ZSB in the moss peat applied as inoculants on seed and left for 2 hours in the laminar flow cabinet for drying and avoid contamination.

### Biochemical and molecular characterization of bacterial strains

Gram staining of the unidentified strains, colony morphology, cell shape, temperature and pH range tests were done according to Aslam et al. [25]. The DNA extraction and purification was done by using Easy-DNA® Kit (Thermo Fisher Scientific). The PCR reactions of 16S rRNA gene were performed using the eubacterial primers 27f (50-AGAGTTTGATCMTGGCTCAG-30) and1492r (50-GGTTACCTTGTTACGACTT-30) from total genomic DNA. The other process from PCR to phylogenetic tree was accomplished by following Aslam et al. [25].

### Planting geometry and crop husbandry

Seedbed was prepared by two-time cultivation followed by planking and ridges were made 75 cm apart with tractor-mounted ridger. Crop was sown in the third week of July by hand-dibblerat P × P distance of 25 cm. Fertilizers were applied @ 250 kg N, 115 kg P and 150 kg K ha^-1^. All the K and P along with one third of N were applied at seedbed preparation, while remaining N was applied in two splits at 3–4 and 6–7 leaf stages. Sources of fertilizers were DAP (Diammonium phosphate), Urea and SOP (Sulphate of potash). Irrigation was done at seven days’ interval from emergence to harvesting except rainfall. For weed control, “Dual Gold 960 EC” (S-Metolachlor) a brand of “Syngenta” was used as pre-emergence herbicide 24 hours after sowing. Carbofuran 3% G was used to avoid stem borer attack.

### Agronomic attributes

Fully matured leaves were collected from each plot and leaf area was recorded by leaf area meter. Cob length was measured with the help of meter rod. Cob diameter was recorded with keen precision by using electronic Vernier calipers. The 100 grains from each plot were weighed on analytical balance to record 100-grain weight.

### Grain yield and biological yield (t ha^-1^)

Three plants from each plot were randomly selected and cobs present on these plants were separated. Grains were separated from cob pith and grain weight was recorded. Crop was harvested at maturity and fresh weight of all plant components (leaves, roots and shoot) was recorded. The harvested plants were dried for 14 days under sunshine and dry weight was recorded. The recorded dry weight was used to compute biological yield.

### Harvest index (HI %)

Harvest index was calculated through dividing the grain yield with biological yield expressed in percentage (%).


$$Harvest\;index=\frac{Grainy\;ield}{Biological\;yield}\times 100$$

### Standards preparation

By using commercially available stock solutions (Applichem®), calibrated standards were prepared (1000 ppm). Working standards were prepared by using highly purified deionized water. All the glass apparatus used in analytical work were immersed in 8N HNO_3_ solution overnight and washed with deionized water before use.

### Zn contents in in leaves, stem cob-pith, roots and grains

The collected samples of different plant parts were dried at 70 ^o^C for 24 hours. Afterwards, Zn concentration was measured by the method of [24]. Briefly, dried grains were ground to fine powder. The 1 g grain flour samples were taken in conical flask of 50 ml and 10 ml concentrated di-acid mixture of (1:2) nitric acid and perchloric acid was added to the flasks and left overnight. After 24 hours, flasks were heated on hot plate at 300 ^o^C until aliquot material became transparent. It was cooled at room temperature and distilled water was added to make 50 ml volume. Zinc in prepared samples was determined by using Atomic Absorption Spectrophotometer (Hitachi Polarized Zeeman AAS, Z-8200, Japan) following the protocol described in AOAC. Instrumental operating conditions were; wavelength = 213.9 nm, slit width = 1.3nm, lamp current = 10 mA, burner height = 7.5 mm, burner head = standard type, flame = Air-C_2_H_2,_ flow rate of oxidant gas pressure = 160 kpa and flow rate of fuel gas pressure = 6 kpa.

### Root measurements

Roots were collected from soil with the help of spade and thoroughly washed. Root length was measured with the help of measuring tape. Root diameter was measured by using digital Vernier caliper. After measuring root length, roots fresh weight was recorded on digital balance. Roots were dried in oven until constant weight. Then dry weight of roots was noted.

### Relative water contents (RWC) %

Relative water contents were determined according to [26]. For the determination of RWC, the flag leaf from the shoot of maize plant was removed with a sharp razor blade. Its fresh weight (fresh mass, FW) was determined immediately. For the determination of turgid weight (TW) leaves were put in the distilled water inside the closed plastic bags. The leaves were allowed for imbibition’s for overnight (24 hours) by placing plastic bags under dim light (around 20 m mol m^2^ s^-1^) in the laboratory under the naturally fluctuating temperature. After the completion of imbibition’s, the leaf samples were again weighed, and turgid weight (TW) was recorded. After recording the turgid weight, the leaf samples were placed at 70°C in an oven for 72 hours. After this, oven-dry weight (DW) of leaf samples was determined. All the measurements were made on an analytical scale, with the precision of 0.0001 g. The RWC was calculated by using the values of FW, TW, and DW by the given equation.


RWC(%)=[(freshweight‐dryweight)/(turgidweight‐dryweight)]*100

### Chlorophyll a and b (mg L^-1^)

Fresh leaf sample were cut into 5 cm small pieces and put in test tubes. The 10 ml 80% acetone solution was poured into each test tube and the tubes were placed at -20°C for 24 h. Test tubes were vortexed for 30 seconds, kept for one hour and then extract was centrifuged at 14000 rpm for 5 minutes at 25°C. Supernatant material was collected and reading was recorded on spectrophotometer at wavelengths of 645 and 663. Chlorophyll a and b contents were calculated by using following equations. Total number of chlorophyll contents was calculated by sum of chlorophyll a and b contents.


$$Chlorophyll\;a\;(mg\;L^{‐1})=12.7\;A_{663}‐2.69\;A_{645}$$

$$Chlorophyll\;b\;(mg\;L^{‐1})=22.9\;A_{645}‐4.68\;A_{663}$$

Here, A663 and A645 represents the absorbance at which values read at 663 and 645 nm wavelengths of spectrophotometer, respectively.

### Electrolyte leakage (%)

Electrolyte leakage (EL) was measured to determine the membrane permeability. Briefly, 1-gram leaf sample was cut into 0.5 cm small pieces. Small pieces were vertically put in test tubes where 10 ml distilled water was added. The tubes were cover with aluminum foil and left at 32°C for four hours. The EC_1_ (dSm^-1^) was recorded with Cond 315i/ Set, WTW Wi~Secnschaftlich-Technische Werkstatton 82362 Weilheim, Germany. The samples were autoclaved for 20 minutes at 121°C. The samples were cooled at room temperature and EC_2_ (dSm^-1^) was recorded. The EL was computed by following formula [27]:

$$EL=EC_{1}/EC_{2}\times 100$$

### Statistical analysis

Statistics 8.1 was used for data analysis. Least significance difference (LSD) test at 5% probability level was used to compare treatment means [28].

## Results and discussion

Cob diameter is very important yield increasing trait, which is significantly improved by priming with Zn-lysine chelate (1.5%) and seed inoculation with ZSB (Table 2). Cob diameter and cob length were increased by 16.75% and 42% during 2016 and by 11.36% and 34.35% during 2017. These results are in agreement with [29]. Proper and timely Zn supply as seed priming and seed inoculation increased Zn uptake in all plant parts. Siddiqui et al. [30] reported that sufficient supply of Zn increased N uptake of maize plants and ultimately increased yield components. Zinc application as seed priming is more important for better productivity as reported by [31]. Similarly, Zn application as seed treatment improved N uptake during milking and grain filling in maize [32].

**Table 2:** Effect of Zn-lysine chelate along with inoculation with consortium of highly Zinc Solubilizing Bacteria on Zn distribution in different parts of maize, grain yield and biological yield.

	2016								
	Cob length (cm)	Cob diameter (mm)	No of grains/row	100 grains weight (g)	Leaf area (cm^2^)	Primary Root length (cm)	Primary root Diameter (mm)	Root fresh weight (g)	Root dry weight (g)
**T**_**0**_	14.33F	45.54E	30.33F	42.83D	645.23H	757.0J	133.66E	77.33G	19.36G
**T**_**1**_	14.56EF	46.17E	33.33E	43.60CD	658.60H	804.9I	136.17E	98.33F	24.60F
**T**_**2**_	15.46DF	48.30D	38.00CD	46.76A-D	725.70G	841.8H	167.74D	119.67E	29.93E
**T**_**3**_	17.13CD	50.44C	39.00B-D	47.40A-C	773.97F	959.6F	186.82C	126.67DE	31.70DE
**T**_**4**_	18.00BC	51.05BC	39.66BC	48.23AB	810.77E	1007.8E	188.16C	135.33CD	33.86B-D
**T**_**5**_	18.33BC	51.32BC	40.33A-C	48.63AB	837.33DE	1032.5D	214.53B	136.33B-D	34.10B-D
**T**_**6**_	16.03DE	48.01D	36.66D	46.03B-D	714.07G	902.5G	190.27C	127.00DE	31.76DE
**T**_**7**_	18.36BC	50.57C	38.66CD	47.50A-C	851.03CD	1014.0E	198.92C	134.67CD	33.66CD
**T**_**8**_	19.10AB	51.27BC	40.66A-C	48.40AB	884.67BC	1070.5C	220.31B	138.00BC	34.53BC
**T**_**9**_	19.33AB	52.53AB	41.66AB	49.83AB	918.87B	1239.5B	240.34A	145.33AB	36.33AB
**T**_**10**_	20.36A	53.17A	43.00A	50.56A	970.97A	1374.3A	249.91A	150.67A	37.700A
LSD =	1.68	1.51	2.75	4.08	36.73	11.64	12.20	9.99	2.50
	2017								
	Cob length (cm)	Cob diameter (mm)	No of grains/row	100 grains weight (g)	Leaf area (cm^2^)	Primary Root length (cm)	Primary root Diameter (mm)	Root fresh weight (g)	Root dry weight (g)
**T**_**0**_	14.96E	46.54E	32.00F	43.48C	655.87H	752.70I	133.99G	80.33G	24.10G
**T**_**1**_	15.56DE	47.84DE	33.66F	43.58C	678.27GH	802.91H	152.17F	96.67F	29.00F
**T**_**2**_	16.80CD	48.64CD	37.00E	46.10A-C	737.03EF	839.10G	174.41E	109.33E	32.80E
**T**_**3**_	17.80BC	50.40AB	38.00DE	46.08A-C	788.30DE	949.90E	186.82DE	125.33D	37.93D
**T**_**4**_	18.66AB	50.88AB	38.66C-E	47.53A-C	805.83D	1022.50D	192.16D	131.33D	39.40D
**T**_**5**_	18.80AB	50.98AB	40.00B-D	47.61A-C	840.67CD	1041.91D	216.36C	143.67C	43.76C
**T**_**6**_	15.70DE	48.35CD	37.33E	44.19BC	729.07FG	901.10F	188.27DE	130.00D	39.67D
**T**_**7**_	18.63AB	49.57BC	38.66C-E	46.50A-C	867.70BC	929.61E	197.92D	147.00C	45.43C
**T**_**8**_	18.86AB	50.61AB	40.33BC	47.71AB	888.00BC	1073.82C	226.65BC	171.33B	51.40B
**T**_**9**_	19.03AB	51.53A	41.66AB	49.16A	918.87AB	1241.20B	238.34AB	177.00AB	53.43B
**T**_**10**_	20.10A	51.83A	42.66A	50.12A	967.63A	1344.30A	248.58A	186.33A	57.57A
LSD =	1.49	1.72	2.29	4.14	53.98	23.71	17.583	11.11	3.06

LSD = Least significant difference, T_0_(Control) = No priming nor inoculation, T_1_ = Hydro-priming, T_2_ = Priming with 0.1% Zn-lysine chelate, T_3_ = Priming with 0.5% Zn-lysine chelate, T_4_ = Priming with 1.0% Zn-lysine chelate, T_5_ = Priming with 1.5% Zn-lysine chelate, T_6_ = Inoculation with consortium of highly ZSB, T_7_ = Priming with 0.1% Zn-lysine chelate + Inoculation with consortium of highly ZSB,T_8_ = Priming with 0.5% Zn-lysine chelate + Inoculation with consortium of highly ZSB,T_9_ = Priming with 1.0% Zn-lysine chelate + Inoculation with consortium of highly ZSB,T_10_ = Priming with 1.5% Zn-lysine chelate + Inoculation with consortium of highly ZSB.

The highest 100-grain weight was recorded for combined application of Zn-lysine chelate as (1.5%) and ZSB inoculation during both years. Higher 100-grain weight might be due to increased cob length and diameter, which produce heavier grains. Increased 100-grain weight, cob length and cob diameter are reported by Tahir et al. [33] with foliar application of Zn. The increase in 100-grain weight over control was 18.4% and 15.27% for 2016 and 2017, respectively. These results are close to the findings of Mohsin et al. [28] where 100-grain weight was improved by 19% through seed priming.

Leaf area is an important factor contributing towards better growth and development of crop. Seed priming along with ZSB inoculation significantly improved leaf area (Table 2). Higher values of leaf area and harvest index might be attributed to increased values of tryptophan amino acid and other growth promoting hormones responsible factor for leaf expansion [34]. Higher leaf area resulted in more leaf area index, crop growth rate and net assimilation rate, which increased dry matter production. Increased leaf area and leaf area index has been reported by Safyan et al. [35] for foliar application of Zn.

Healthy root system is an important characteristic for healthy plant growth and development. Zinc application significantly enhanced total number of roots per plant, root length, root diameter. Hence, plants had more root surface area, which enabled them to absorb more water and nutrients from rhizosphere. Increased total root length and root diameter observed for Zn seed priming along with ZSB inoculation (Table 2). Increase in the root length and diameter was due to better Zn nutrition at early growth stages as reported by [24]. Hafeez et al. [36] reported positive effect of ZSB on plant growth as compared to control treatment.

Application of Zn through seed priming with Zn-lysine chelate along with ZSB inoculation significantly improved Zn contents in all plant parts during both years (Table 3). The Zn contents were significantly increased in all the parts; however, the highest Zn contents were recorded during 2017 with seed priming (1.5% Zn-lysine chelate) and ZSB inoculation. The Zn contents were increased by 15.3%, 15.6%, 49.1%, and 33.0% in grain, cob-pith, stem and roots, respectively compared from control. Increased Zn contents in all the plant parts might be due to timely provision of Zn as seed priming [28]. The prominent increase in Zn contents in all the plant parts is also reported by [28, 37].

**Table 3:** Effect of Zn lysine chelate priming and inoculation of ZSB on agronomic traits of maize.

Zn +ZSB	2016						
	Zn in Grain (ppm)	Zn in stem (ppm)	Zn in Leaves (ppm)	Zn in cob-pith (ppm)	Zn in roots (ppm)	Grain Yield t/ha	Biological Yield t/ha
**T**_**0**_	7.10 E	3.20 F	4.10 F	3.93 F	3.86 D	11.39 F	16.91 G
**T**_**1**_	7.16 DE	3.40 EF	4.83 EF	4.23 F	3.93 D	12.14 F	17.30 FG
**T**_**2**_	7.43 C-E	3.63 EF	5.76 DE	4.40 EF	4.36 CD	12.88 EF	17.90 F
**T**_**3**_	7.63 B-E	3.86 EF	6.06 CD	4.76 EF	4.56 B-D	14.68 CD	18.80 E
**T**_**4**_	7.73 A-D	4.00 EF	6.13 CD	5.10 DE	4.60 B-D	15.23 A-D	19.28 DE
**T**_**5**_	7.76 A-C	4.43 E	6.20 B-D	6.00 C	5.20 AB	16.11 A-C	20.04 D
**T**_**6**_	7.23 C-E	3.90 EF	6.63 B-D	5.80 CD	4.33 CD	13.79 DE	18.83 E
**T**_**7**_	8.13 AB	6.83 D	6.80 BC	6.30 C	4.46 B-D	15.09 B-D	19.22 E
**T**_**8**_	8.13 AB	8.23 C	7.13 B	6.43 BC	4.63 A-D	15.89 A-C	21.27 C
**T**_**9**_	8.20 AB	10.63 B	7.16 B	7.16 B	4.80 A-C	16.23 AB	22.47 B
**T**_**10**_	8.23 A	13.16 A	9.80 A	8.20 A	5.40 A	16.64 A	23.41 A
LSD =	0.59	1.16	0.98	0.84	0.78	1.49	0.78
Zn +ZSB	2017						
	Zn in Grain (ppm)	Zn in stem (ppm)	Zn in Leaves (ppm)	Zn in cob-pith (ppm)	Zn in roots (ppm)	Grain Yield t/ha	Biological Yield t/ha
**T**_**0**_	7.03E	3.23E	4.00E	4.00F	4.00C	11.19 D	16.083 G
**T**_**1**_	7.03E	3.66DE	5.50D	4.00F	4.13C	11.61 D	16.25 G
**T**_**2**_	7.46CE	3.60DE	6.00CD	4.23EF	4.53BC	13.46 C	16.74 FG
**T**_**3**_	7.50CE	3.83DE	6.00CD	4.70EF	4.50BC	14.42 A-C	17.81 E
**T**_**4**_	7.60C-E	3.96DE	6.00CD	5.06DE	4.50BC	14.76 A-C	19.12 D
**T**_**5**_	7.70B-D	4.33DE	6.00CD	6.03C	5.00AB	15.40 AB	20.10 C
**T**_**6**_	7.30DE	4.60D	6.50BC	5.83CD	4.50BC	14.18 BC	17.48 EF
**T**_**7**_	7.80A-D	6.66C	6.66BC	6.00C	4.50BC	15.41 AB	18.88 D
**T**_**8**_	7.96A-C	8.30B	7.03B	6.46BC	4.50BC	15.87 AB	20.59 BC
**T**_**9**_	8.23AB	9.10B	7.00B	7.06B	4.50BC	15.89 A	21.39 B
**T**_**10**_	8.30A	13.83A	10.50A	8.33A	5.50A	16.06 A	23.69 A
LSD =	0.57	1.27	0.85	0.87	0.79	1.72	0.89

LSD = Least significant difference, T_0_(Control) = No priming nor inoculation, T_1_ = Hydro-priming, T_2_ = Priming with 0.1% Zn-lysine chelate, T_3_ = Priming with 0.5% Zn-lysine chelate, T_4_ = Priming with 1.0% Zn-lysine chelate, T_5_ = Priming with 1.5% Zn-lysine chelate, T_6_ = Inoculation with consortium of highly ZSB, T_7_ = Priming with 0.1% Zn-lysine chelate + Inoculation with consortium of highly ZSB, T_8_ = Priming with 0.5% Zn-lysine chelate + Inoculation with consortium of highly ZSB, T_9_ = Priming with 1.0% Zn-lysine chelate + Inoculation with consortium of highly ZSB, T_10_ = Priming with 1.5% Zn-lysine chelate + Inoculation with consortium of highly ZSB. ppm = parts per million (μg/g); t/ha = tones/hectare.

Seed priming and ZSB inoculation improved grain and biological yields during both years. Increased grain and biological yield are the result of adequate and proper Zn supply, which increased cob length, cob diameter, grains per cob and 100 grains weight. Enhanced carbohydrates synthesis and translocation towards grain are the possible reasons behind improved grain and biological yield [38, 39]. Improved biological yield might be due to proper and better nutrition at early stages, which improved early growth of plants and increased dry matter production. Biological yield was increased due to increased leaf area and more plant height [40]. In the same way, Trehan and Sharma [41] reported increased dry matter production with Zn application for maize crop. In addition, Zn also improved harvest index. Plant growth promoting and Zn solubilizing activities of microorganisms (fungi and bacteria) had significant results on Zn solubilization in Shakeel et al. [42] Greater values of biological yield might be due to better crop nutrition provided by Zn seed priming which enhanced N uptake. In the same way, Trehan and Sharma [40] revealed that Zn application increased dry matter production of maize hybrids. Higher values of biological yield might be due to increase in plant height and healthy leaves [33].

Higher values of Electrolyte leakage (EL) in maize leaves were recorded in control treatment during both years (Table 4). On the other hand, decreased values of EL was observed for 1.5% Zn application as seed priming along with ZSB inoculation. A 57% and 56% reduction in EL was observed for 1.5% Zn + ZSB inoculation, whereas 40% and 52% reduction was recorded for 1.5% Zn application during 2016 and 2017, respectively. Higher values of EL are due to more membrane damage, whereas Zn application provided more strength to the membrane and caused less damage. Zinc application improved membrane integrity and decreased membrane damage. Proper Zn nutrition ameliorated EL with lower values than control treatments. Shakeel et al. [42] observed that reduction in growth could alter the levels of endogenous hormones and these hormonal regulations are involved in membrane permeability and water relations. Increased relative water content was observed in T_10_ (Table 4) as compared to control treatment during 2016 and 2017.

**Table 4:** Effect of Zn lysine chelate priming and inoculation of ZSB on biochemical traits and water relations of maize plants.

	2016					
	30 DAE		At Maturity			
	Chlorophyll-a	Chlorophyll-b	Chlorophyll-a	Chlorophyll-b	EL (%)	
**T**_**0**_	16.76D	35.40F	12.80E	22.40F	74.057A	44.26F
**T**_**1**_	20.16B-D	36.36EF	13.63DE	24.23EF	74.000A	44.93EF
**T**_**2**_	20.63B-D	38.93D-F	16.20A-D	28.03CD	69.473A	50.96D-F
**T**_**3**_	20.30B-D	40.46CD	16.10B-D	29.63B-D	58.620B	52.46D
**T**_**4**_	22.90AB	41.43B-D	16.46A-C	30.56A-C	48.173C	54.43CD
**T**_**5**_	22.43A-C	43.40BC	17.60A-C	30.16B-D	44.050C	58.16CD
**T**_**6**_	18.86CD	39.40DE	15.10C-E	27.10DE	58.130B	51.60DE
**T**_**7**_	20.90A-C	44.53AB	16.70A-C	31.36AB	46.370C	61.63BC
**T**_**8**_	22.86A-C	44.86AB	17.10A-C	32.63AB	41.043CD	68.30AB
**T**_**9**_	23.76AB	45.00AB	18.20AB	33.40A	35.953DE	70.80A
**T**_**10**_	24.70A	47.60A	18.83A	33.63A	31.470E	73.93A
LSD =	4.01	3.96	2.70	3.21	7.55	7.32
	2017					
	30 DAE		At Maturity			
	Chlorophyll-a	Chlorophyll-b	Chlorophyll-a	Chlorophyll-b	EL (%)	RWC (%)
**T**_**0**_	17.33E	36.63G	13.67E	22.87E	73.39A	46.30F
**T**_**1**_	19.83C-E	37.63G	14.30DE	23.90E	66.34A	48.93EF
**T**_**2**_	20.30CD	39.60F	15.53CD	27.70D	55.11B	52.96D-F
**T**_**3**_	20.20CD	41.13DE	15.70CD	29.30B-D	46.21CD	53.76D-F
**T**_**4**_	20.23CD	42.20CD	16.23C	29.90B-D	34.50F	58.15CD
**T**_**5**_	20.50B-D	43.50BC	16.60BC	30.50A-D	51.13BC	58.15CD
**T**_**6**_	19.53DE	39.70EF	14.77DE	28.77CD	69.38A	57.25C-E
**T**_**7**_	22.56A-C	43.20BC	16.37C	30.70A-C	43.03DE	60.61B-D
**T**_**8**_	21.53A-D	44.20B	16.53BC	31.70 AB	38.04EF	64.61A-C
**T**_**9**_	23.10AB	44.33B	17.87AB	31.93AB	36.62EF	67.45AB
**T**_**10**_	24.03A	45.93A	18.07A	32.87A	32.13F	72.94A
LSD =	2.75	1.48	1.42	2.84	8.07	8.73

LSD = Least significant difference, T_0_(Control) = No priming nor inoculation, T_1_ = Hydro-priming, T_2_ = Priming with 0.1% Zn-lysine chelate, T_3_ = Priming with 0.5% Zn-lysine chelate, T_4_ = Priming with 1.0% Zn-lysine chelate, T_5_ = Priming with 1.5% Zn-lysine chelate, T_6_ = Inoculation with consortium of highly ZSB, T_7_ = Priming with 0.1% Zn-lysine chelate + Inoculation with consortium of highly ZSB, T_8_ = Priming with 0.5% Zn-lysine chelate + Inoculation with consortium of highly ZSB, T_9_ = Priming with 1.0% Zn-lysine chelate + Inoculation with consortium of highly ZSB, T_10_ = Priming with 1.5% Zn-lysine chelate + Inoculation with consortium of highly ZSB. ppm = parts per million (μg/g); t/ha = tones/hectare. EL = Electrolyte leakage, RWC = Relative water contents.

The ZSB were identified by BLAST in NCBI data using 16S rRNA gene sequencing data. The four strains PMEL-1, PMEL-48, PMEL-57 and PMEL-71 were identified as species of genera *Alcaligenes* sp., *Bacillus* sp., *Pseudomonas* sp. and *Bacillus* sp., respectively (Fig 1, Table 5). The consortium of these strains played very active role in Zn-solubilizing and effectively uptake in plants as shown in Table 3. The maximum uptake and translocation was observed when 1.5% Zn-lysine chelate and consortium of highly ZSB [43, 44].

**Fig 1:** Phylogenetic tree constructed from comparative analysis of 16S rRNA gene sequences showing the relationships between strains PMEL-1, PMEL-48, PMEL-57 and PMEL-71 and their related species of different genera (Table 5). The tree was constructed by using the neighbour-joining method and Jukes & Cantor evolutionary distance matrix data obtained from aligned nucleotides. Bootstrap values (expressed as percentage of 1000 replications) greater than 50% are shown at the branch points. Bar, 1 substitution per 100 nucleotide positions.

**Table 5:** Identification of bacterial strains from BLAST on the basis of 16S rRNA gene sequencing and their similarity with type strains.

Strain name	bp	Similarity %	Top-hit taxon	Top-hit taxonomy
PMEL-1	1464	99.22	*Alcaligenesfaecalis* subsp. Parafaecalis G^T^	Bacteria;Proteobacteria;Betaproteobacteria;Burkholderiales;Alcaligenaceae;Alcaligenes;Alcaligenes faecalis
PMEL-48	1469	100%	*Bacillus cereus* ATCC 14579^T^	Bacteria;Firmicutes;Bacilli;Bacillales;Bacillaceae;Bacillus
PMEL-57	1453	96.96	*Pseudomonas marginalis* ATCC 10844^T^	Bacteria;Proteobacteria;Gammaproteobacteria;Pseudomonadales;Pseudomonadaceae;Pseudomonas
PMEL-71	1471	99.73	*Bacillus cereus* ATCC 14579^T^	Bacteria;Firmicutes;Bacilli;Bacillales;Bacillaceae;Bacillus

## Conclusion

It can be concluded from this experiment that seed priming with 1.5% Zn-lysine chelate in combination with ZSB inoculation significantly improved cob diameter and cob length by 16.75% and 42% during 2016 and by 11.36% and 34.35% during 2017. The increase in 100 grains weight over control was 18.4% and 15.27% for 2016 and 2017, respectively. The Zn contents were increased by 15.3%, 15.6%, 49.1%, and 33.0% in grain, cob-pith, stem and roots, respectively compared from control. Thus, combination of 1.5% Zn-lysine chelates and ZSB inoculation could be used for combating malnutrition.
